# Prevalence, Predictors, and Clinical Presentation of Acute Pericardial Effusion Following Percutaneous Coronary Intervention

This article has been retracted.

**DOI:** 10.3389/fcvm.2021.759164

**Published:** 2022-01-11

**Authors:** Bei Zhao, Jie Zhang, Yun Li, Xueyao Feng, Shuai Mao, Zhao Yin, Li Liu, Dapeng Song, Shouli Wang

**Affiliations:** ^1^Department of Cardiology, People's Liberation Army Strategic Support Force Characteristic Medical Center, Beijing, China; ^2^Outpatient Department, The 22nd Retirement Home for Resigning Cadres in Haidian District, Beijing Garrison of People's Liberation Army, Beijing, China

**Keywords:** pericardial effusion (PE), percutaneous coronary intervention, post-cardiac injury syndrome, non-STEMI, unstable angina (UA), stable angina

## Abstract

**Background:** Iatrogenic pericardial effusion (PE) has been demonstrated to lead to cardiac injury as a sign of systemic inflammatory response.

**Objectives:** This study sought to determine the anatomical characteristics and clinical presentation associated with PE after percutaneous coronary intervention (PCI) by using echocardiography.

**Methods:** The clinical outcomes of all patients with coronary artery disease who underwent PCI from July 2014 to December 2018 were evaluated. The quantitative and qualitative analyses of PE were performed. The associations between the presence of PE and procedural factors were also evaluated.

**Results:** A total of 882 patients were enrolled. PE was found in 144 patients (16.3%) and was mostly located in the anterior pericardium at low amounts. The serum levels of high-sensitive C-reaction protein before PCI and troponin T in the group with PE after PCI were significantly higher than those in the group without PE (*p* < 0.0001). The presence of PE was associated with the procedural time (OR = 1.02, *p* = 0.035) and the degree of interventional complexity (multiple vessels OR = 1.89, *p* = 0.014; chronic total occlusion OR = 2.04, *p* = 0.005; and PCI with rotational atherectomy OR = 1.15, *p* = 0.011) independent of the number of culprit vessels and stents. During 1-year follow-up, a significantly higher number of cardiac deaths (3) and myocardial infarctions (8) occurred in patients with PE than in patients without PE (*P* < 0.05).

**Conclusion:** Post-PCI acute PE was frequent, generally mild, mainly asymptomatic, and independently associated with procedural time and complexity. This effusion, which is considered as a cardiac damage marker, could be a predominant clinical sign for long-term prognosis.

## Introduction

Pericardial effusion (PE) can develop from any condition that affects the pericardium, including pericarditis and a variety of systemic disorders (1, 2). In addition, PE may have important implications for disease prognosis or diagnosis. The clinical causes of PE are very diverse; iatrogenic causes, in addition to common causes, such as infections, malignancies, and autoimmune or idiopathic diseases, have attracted attention (3, 4). In particular, cardiac injuries induced by cardiac surgery or myocardial infarction, which are also known as post-cardiac injury syndrome (PCIS) and Dressler's syndrome, have been observed (5, 6). Interventional cardiology procedures with less trauma than open cardiovascular surgery are increasingly performed nowadays. Interestingly, the signs of a systemic inflammatory response have also been observed after interventions, such as the implantation of stents, aortic stent-grafts, aortic valves, and heart rhythm devices and radiofrequency ablation (7). A few reports have recently described PCIS as a complication of endovascular procedures, such as percutaneous cardiac intervention (8). However, until now, the clinical presentation of PE in the stent area following percutaneous coronary intervention (PCI) has been poorly evaluated. Thus, the aim of this study was to evaluate the prevalence and clinical characteristics of PE and the relationship of PE with procedural factors to investigate its long-term prognosis.

## Methods

### Study Population

This work was a single-center retrospective observational study performed at PLA Strategic Support Force Characteristic Medical Center (Beijing 306 Hospital), Beijing, China. We evaluated 914 patients with *de novo* coronary artery disease who required PCI staging from July 2014 to December 2018. Forty-nine patients were excluded due to the reasons listed in Figure 1. Patients of STEMI undergoing emergency PCI were excluded because most lacked the time for echocardiography examination before the procedure. For the purpose of the study, only patients with post-procedural PE were included. Patients with pre-procedural PE for any cause were also excluded. Consequently, 882 patients were included, of whom 554 presented with non-STEMI (NSTEMI, 194) and unstable angina (360) and 328 presented with stable angina.

**Figure 1:** Flow chart of the study.

### Echocardiography

All enrolled patients underwent transthoracic echocardiography (TTE) with PHILIPS IE Elite (Netherlands) to identify PE at the pre- and post-procedural stages. The post-procedural change in PE was assessed after the index procedure in 2 h and at 72 h after hospital admission. A generally accepted system for grading effusions as minimal, mild, moderate, or large was provided by the 2015 ESC guidelines (9). Any PE with <5 mm of pericardial separation in diastole was defined as minimal. A PE with a separation of 5 mm to 10 mm was graded as mild. A PE with a separation of 10 mm to 20 mm was graded as moderate. A PE with a separation >20 mm was graded as large. Patients were divided into two groups in accordance with the absence or presence of PE after the index procedure. The group without PE was defined on the basis of a pericardial separation of <4 mm before the procedure and normal thickness of usually 1–2 mm in diastole. Hemodynamically significant PE was defined as respiratory variation of mitral inflow ≥25% with the existence of inferior vena cava plethora (inspiratory diameter collapse <50%) and the diastolic collapse of the right atrium or ventricle. PE was assessed from standard TTE by using the parasternal long-axis, short-axis, four-chambers, and subcostal views and was quantified during diastolic timing by using the M mode on the posterior wall. PE at the anterior pericardium was evaluated from the anterior wall before the right ventricle from the parasternal long-axis view and confirmed from the subcostal views. The posterior pericardium was determined from the posterior wall behind the left ventricle from the parasternal long-axis view. Echocardiography data before and after the procedure were compared to differentiate PE from pericardial fat. The diagnosis of epicardial fat tissue was retained if the echo-free space was located anteriorly, tended to move in concert with the heart, and remained stable as determined through the comparison of the echocardiography data taken before and after the procedure. PE associated with PCI was diagnosed when PE occurred after PCI and other possible causes, such as acute STEMI, congestive heart failure, renal disease, hypothyroidism, and idiopathic PE, were excluded. The echocardiography examination was performed on all patients by one special echocardiography doctor, and the results were reviewed and confirmed by two echocardiography experts. The patients were followed up at 1, 3, and 12 months with 12-lead ECG and echocardiography.

### Procedures

PCI was carried out in the usual manner after the administration of dual antiplatelet therapy (DAPT, aspirin/clopidogrel) and unfractionated heparin. DES was deployed from the normal-to-normal segment as evaluated by angiography or intravascular imaging. Multivessel disease was defined as double or triple vessels that were implanted with stents. Bifurcation disease was described as bifurcation lesions with at least two stents by using the Culotte or Crush model. Chronic total occlusion (CTO) and rotational atherectomy (RA) were defined as the complex procedure. Patients continued to take DAPT (100 mg aspirin and 75 mg clopidogrel) daily for 12 months then were placed on aspirin monotherapy indefinitely.

### Study Endpoints

The primary study endpoint was the presence of PE after the index procedure. The secondary study endpoints included (1) changes in PE at different time points; (2) major adverse cardiac–cerebral events (MACCEs) up to 12 months of clinical follow-up. MACCEs included all-cause death, cardiac death, myocardial infarction, heart failure, and stroke.

### Statistical Analysis

The normality of the data was verified by using the Kolmogorov–Smirnov test because most values were not normally distributed. Continuous variables were expressed as mean ± SD along with median values (first and third quartiles). Univariate comparison between patients with and without PE was performed by using Mann–Whitney *U* test and *t* test for continuous variables. Categorical data were expressed as frequencies and compared by using the *χ*^2^ test or Fisher's exact test as appropriate. The relationship between PE and procedural factors was assessed with a multivariable logistic regression model along with the known clinical risk factors. Data analysis was performed by applying SPSS 25 (IBM, Beijing, China). Here, *p* < 0.05 was considered statistically significant.

## Results

### Study Population

A total of 882 consecutive patients (mean age 62.5 ± 11.9 years, 23.1% female) were enrolled. A total of 144 patients (16.3%) had PE after the index procedure. They included 85 patients with stable angina and 59 patients (33.4%) with unstable angina or NSTEMI. The baseline clinical and procedural characteristics of the study population are detailed in Tables 1, 2. Among the patients, 70.8% had single-vessel disease (38.4, 10.8, and 21.6% of the culprit lesions were located in the left anterior descending artery, left circumflex artery, and right coronary artery, respectively). Multivessel disease accounted for 14.8% of the cases. The percentages of CTO and RA in complex procedures were 12.5 and 9.3%, respectively. Comparing the groups with and without PE revealed that the patients' baseline and vessel characteristics were not significantly different. The patients with PE had significantly longer total procedural time (196.6 ± 98.4 min vs. 151.4 ± 94.5 min, *p* = 0.001) and fluoroscopy time (48.6 ± 11.2 min vs. 42.4 ± 12.3 min, *p* = 0.014) than the patients without PE. The maximum PE size in the PE group was significantly higher than that in the group without PE (6.09 ± 3.33 mm vs. 1.63 ± 1.14 mm, *p* < 0.0001).

**Table 1:** Baseline clinical characteristics.

**Variable**	**All patients** **(***n*** =882)**	**Patients without PE** **(*n* = 738)**	**Patients with PE** **(***n*** = 144)**	***P*** **-value**
Age (year)	62.5 (51.0, 74.0)	63.4 (52.0, 75.0)	62.1 (50.0, 73.0)	0.06
Female (%)	23.1 (204)	25.3 (187)	21.6 (31)	0.06
Body mass index (kg/m^2^)	30.1 (22.3, 37.9)	29.5 (21.1, 36.5)	30.5 (21.6, 39.8)	0.29
Diabetes mellitus	33.4 (295)	35.3 (261)	32.2 (46)	0.09
Hypertension	47.3 (417)	49.5 (365)	46.2 (67)	0.05
Hyperlipidemia	61.7 (544)	59.5 (493)	62.4 (90)	0.16
Current Smoking	19.3 (170)	15.4 (114)	23.8 (34)	0.03
Previous myocardial infarction	17.7 (156)	18.2 (134)	22.1 (32)	0.17
Previous PCI	32.6 (288)	33.4 (246)	29.7 (43)	0.38
Previous CABG	11.1 (98)	12.1 (89)	9.2 (13)	0.52
Baseline LDL mmol/L	2.7 (2.2, 3.2)	2.6 (2.1, 3.1)	2.8 (2.2, 3.3)	0.26
Usage of statin at admission	73.4 (647)	72.8 (537)	69.3 (100)	0.67
Stable angina	62.4 (550)	63.6 (469)	59.3 (85)	0.32
NSTEMI and unstable angina	37.6 (332)	36.4 (269)	40.7 (59)	0.51

*CABG, coronary artery bypass grafting; PCI, percutaneous coronary intervention; STEMI, ST-segment elevation myocardial infarction; PCI, percutaneous coronary intervention*.

**Table 2:** Baseline vessels and procedural characteristics.

**Variable**	**All patients** **(***n*** = 882)**	**Patients without PE** **(***n*** = 738)**	**Patients with PE** **(***n*** = 144)**	***P*** **-value**
LM	3.1 (27)	3.2 (24)	3.0 (4)	0.09
LAD	38.4 (339)	40.4 (298)	37.2 (54)	0.08
LCX	10.8 (95)	11.5 (85)	10.5 (15)	0.1
RCA	21.6 (191)	22.8 (168)	20.2 (29)	0.14
Multi-vessel disease	14.8 (131)	12.7 (94)	15.9 (23)	0.05
CTO	12.5 (112)	11.3 (83)	15.4 (22)	0.02
Bifurcation disease	6.8 (60)	7.1 (52)	6.4 (9)	0.59
PCI with RA	9.3 (82)	8.1 (60)	12.7 (18)	0.01
Successful procedure	97.2 (857)	97.8 (722)	96.6 (139)	0.42
Procedural time (min)	177.9 (98.2, 257.6)	151.4 (71.6, 231.2)	196.6 (102.4, 290.8)	0.001
Fluoroscopy time (min)	43.2 (22.4, 64.1)	42.4 (20.7, 64.1)	48.6 (26.3, 70.9)	0.014
Contrast volume (ml)	242.5 (123.5, 393.7)	240.4 (108.8, 372)	258.6 (123.5, 393.7)	0.021
Number of stents	2.22 (1.8, 2.64)	2.21 (1.8, 2.62)	2.28 (1.9, 2.63)	0.35
EF% at admission	51.5 (46.7, 56.3)	50.9 (44.3, 57.5)	51.6 (46.1, 57.1)	0.64
Maximum PE size (mm)	3.86 (1.8, 5.3)	1.63 (0, 2.23)	6.09 (4.6, 5.9)	<0.0001

*CTO, chronic total occlusion; LAD, center anterior descending coronary artery; LCX, center circumflex coronary artery; PCI, percutaneous coronary intervention; RCA, right coronary artery; MI, myocardial infarction; RA, Rotational Atherectomy*.

### Characteristic of PEs

Either the diffused or circumferential echo-free effusion dimensions may differ in the views examined. In all 144 patients, hemodynamically significant PE was found only in two patients with NSTEMI for subacute cardiac rupture. Moderate PE was found in four patients, including three patients with CTO perforation and one patient with post-procedural pericarditis. Most of the post-procedural PEs were mild. Effusions over the anterior and posterior pericardium were frequently evident irrespective of the culprit vessels and disease type (Figure 2). Only three patients out of the 144 patients (2%) complained of pericarditis pain associated with PE. These patients were treated with non-steroidal anti-inflammatory drugs. None of these patients had tamponade or required surgical evacuation. PE was self-limiting in all of these patients given that almost all of the patients had no PE on the TTE performed 1 month after the index procedure (6.09 ± 3.33 vs. 3.39 ± 2.39, *p* < 0.0001). No significant differences were observed in PEs at 72 h after admission and the index procedure (5.83 ± 3.21 vs. 3.39 ± 2.39, *p* = 0.56) (Figure 3).

**Figure 2:** Relationship between PE distribution and culprit vessels in patients with PE.

**Figure 3:** Change of PE at different follow up time point.

### Characteristics of Patients With or Without PE

As shown in Figure 4, the plasma high-sensitive C-reaction protein (hs-CRP, normal range: 0–5 mg/L) level before PCI was significantly higher in patients with PE than in patients without PE (5.16 ± 6.61 vs. 2.95 ± 3.27, *p* < 0.001). Post-PCI troponin T (TnT, normal range: 0–26 pg/ml) level was also significantly higher in patients with PE than in patients without PE (1.77 ± 6.13 vs. 0.44 ± 1.59, *p* < 0.001). These results indicated that the generation of PE following PCI was related to the cardiac inflammatory response.

**Figure 4:** Expression of hs-CRP and TnT in patients with or without PE.

### Association Between Procedural Factors and PE Presence

Multivariable logistic regression was performed by adjusting for the following risk factors: age, sex, currently smoking, diabetes mellitus, hypertension, hyperlipidemia, prior myocardial infarction, prior PCI, prior CABG, baseline LDL, and statin (Table 3). For procedural factors, total procedural time was positively correlated with the presence of PE (OR = 1.02, *p* = 0.035), whereas total fluoroscopy time and contrast volume were unrelated to PE. For procedural complexity, multiple vessels, CTO, and RA were significantly associated with the presence of PE (OR = 1.89, *p* = 0.014; OR = 2.04, *p* = 0.005 and OR = 1.15, *p* = 0.011). The trend of long procedural time and highly complex procedural type was observed in patients with PE. Typical cases were showed in Figure 5.

**Table 3:** Association between procedural factors and presence of PE.

**Endpoint**	**Independent variable**	**OR (95% CI)**	***P*** **-Value**
**Procedural factors**			
	Procedural time	1.02 (1.01, 1.13)	0.035
	Fluoroscopy time	1.00 (0.94, 1.07)	0.990
	Contrast volume	1.00 (0.99, 1.02)	0.389
	Number of stents	1.33 (0.84, 1.79)	0.100
**Procedure complexity**			
	Multiple vessel	1.89 (1.36, 3.11)	0.014
	Bifurcation with two-stent	1.87 (0.39, 2.94)	0.250
	CTO	2.04 (1.47, 3.82)	0.005
	PCI with RA	1.15 (1.04, 2.33)	0.011

*RA, Rotational atherectomy; CTO, chronic total occlusion*.

**Figure 5:** 

### MACCE Endpoints

MACCE rates and components are listed in Table 4. One-year MACCE tended to be higher in patients with PE than in patients without PE. The cardiac death rate was higher in patients with PE (2.8%) than in patients without PE (0.4%). MI and TLR/TVR were significantly higher in patients with PE than in those without PE.

**Table 4:** Major adverse cardio-cerebral events in all patients for 1 year follow-up.

	**All patients** **(***n*** = 882)**	**Patients** **without PE** **(***n*** = 738)**	**Patients** **with PE** **(***n*** = 144)**	***P*** **-value**
Cardiac death	0.8 (7)	0.4 (3)	2.1 (4)	0.02
TLR/TVR	3.0 (26)	2.3 (17)	6.3 (9)	0.02
Stroke	0.7 (6)	0.4 (3)	2.1 (3)	0.09
MI	2.5 (22)	1.9 (14)	5.6 (8)	0.02
Stent thrombosis	0.2 (2)	0.3 (2)	0 (0)	0.75
Total	7.1 (63)	5.7 (42)	14.6 (21)	0.0002

*MI, myocardial infarction; TLR, target lesion revascularization; TVR, target vessel revascularization*.

## Discussion

To the best of our knowledge, this is the first systematic study to evaluate the prevalence and clinical presentation of PE associated with PCI and the effect of PE on clinical prognosis. The main findings of the study were as follows: (1) post-PCI PE was found in 16.3% of the patients irrespective of clinical characteristics. (2) PCI-related PE was generally mild and did not cause symptoms and was more frequently located in the anterior pericardium than in other sites. (3) The presence of PE following PCI was associated with procedural time and interventional complexity degree and was independent of the numbers of culprit vessels and stents. (4) Post-PCI PE was considered as a sign of myocardial injury or cardiac inflammatory response as a interventional complication. (5) PE associated with PCI could persist for several weeks and predict adverse events in the future.

In our study, post-PCI PE most commonly occurred after complex PCI or possibly procedures with long times irrespective of the numbers of culprit vessels and stents. Troughton et al. (10) reported that pericardial complications occur infrequently after percutaneous interventions (11, 12). However, the present work showed that 16.3% of patients had PE following PCI. This value was somewhat higher than previously reported values. Notably, neither of the previous studies specifically looked for PE following PCI and therefore would not have recorded mild, asymptomatic PEs. Our study focused on several issues that were not evaluated in previous studies. Most pericardial effusions can be safely managed with an echo-guided percutaneous approach. In a recent study, only six patients (4.2%) had moderate-to-severe PE for special reasons, such as subacute cardiac rupture, coronary perforation (13). However, most PEs in the study were mild, mainly asymptomatic, and always recovered within 1 month of the index procedure.

The pathophysiology of mild PEs following PCI is unknown. However, histopathological evidence of myocardial damage, including important local inflammatory responses following interventional therapy, has been found in animal models (14) and human hearts (15). Therefore, one possible mechanism could be the inflammation of the pericardium as a result of systemic inflammatory response syndrome, which is an inflammatory activation process that affects the whole body in response to infection or a non-infectious insult, such as trauma, burns, or surgery (16). Interestingly, the signs of a systemic inflammatory response have also been observed after the implantation of stents. This response has the specific name of post-cardiac injury syndrome (PCIS) (17). In our study, the level of plasma hs-CRP before PCI was significantly higher in patients with PE than in patients without PE and corresponded with the elevation of TnT, both measures reflect myocardial involvement and inflammatory status. However, the acute generation of PEs is thought to be due to the early presentation of PCIS, which is believed to be secondary to an autoimmune phenomenon (18). The hypothesized pathophysiology is that the primary injury releases pericardial antigens into the circulation. This phenomenon stimulates an immune response involving the pericardium. Setoyama et al. (19) ascribed the rapid onset of PCIS to the prior stimulation of the immune system by a recent myocardial injury. Even minor injuries that occur at a later time after pre-exposure may trigger the creation of immune complexes and the early activation of the inflammatory pathway. This situation could be another reasonable explanation for the presence of acute PEs in addition to the association of PCI with the total procedural time (OR = 0.98, *p* = 0.035) and interventional complexity (CTO OR = 0.49, *p* = 0.005 and RA OR = 0.87, *p* = 0.011). Long procedural times and highly complicated cases or both should be considered as triggers of procedure-related endothelial, myocardial, or pericardial injuries.

Another possible mechanism of PEs could be correlated to coronary microperforation or subintermal dissection in complicated cases. PCIS after PCI is most frequently described in cases that are complicated by either coronary perforation or dissection (20). In this study, the percentages of CTO and RA in patients with PEs were 12.5 and 9.3%, respectively, which were higher than those in patients without PE. Gabby et al. (21) explained that the initial chest pain caused by PE could have been due to the presence of blood in the pericardium from an aggressive subintimal dissection and microtrauma with knuckle wire. An alternative hypothesis suggests that the leakage of blood into the pericardial space causes PCIS (5, 22). Overall, irritant inflammatory cardiac injury is an emerging cause of PE.

Some studies have demonstrated that moderate and large effusions are likely associated with poor clinical outcome, whereas mild effusions have been related to good overall prognosis (23, 24). The results of our study, which were supported by the results of Mitiku (25), could suggest that the presence of PE following PCI was associated with an increased risk of adverse events and mortality independent of the amount of effusion. Only a large amount of PE is likely based on specific causes. Therefore, the prevalence of PE in patients undergoing PCI in the general population is not negligible. The occurrence of acute PEs suggests the concomitant importance of direct trauma to either the pericardium or the myocardium.

## Limitations

This work was a single-center study with a small sample, and our results need confirmation with a large population of patients. We did not assess the indexes of systemic inflammatory activation, such as hs-CRP and WBC measurements, in later follow-up. The correlation between PEs following PCI and PCIS needs to be further explored.

## Conclusions

Post-PCI acute PE was frequent, generally mild, mainly asymptomatic, and independently associated with procedural time and complexity. Effusion, which was considered as a cardiac damage marker, could be a predominant (OR = 1.89, *p* = 0.014) clinical sign for long-term prognosis.

## Data Availability Statement

The original contributions presented in the study are included in the article/supplementary material, further inquiries can be directed to the corresponding author/s.

## Ethics Statement

The studies involving human participants were reviewed and approved by the Ethics Committee of the PLA Strategic Support Force Characteristic Medical Center. The patients/participants provided their written informed consent to participate in this study. Written informed consent was obtained from the individual(s) for the publication of any potentially identifiable images or data included in this article.

## Author Contributions

BZ and SW: conception and design. SW: administrative support. YL: provision of study materials or patients. JZ, XF, and LL: collection and assembly of data. SM, ZY, and DS: data analysis and interpretation. All authors: manuscript writing and final approval of manuscript.

## Funding

This work was supported by the PLA Strategic Support Force Characteristic Medical Center.

## Conflict of Interest

The authors declare that the research was conducted in the absence of any commercial or financial relationships that could be construed as a potential conflict of interest.

## Publisher's Note

All claims expressed in this article are solely those of the authors and do not necessarily represent those of their affiliated organizations, or those of the publisher, the editors and the reviewers. Any product that may be evaluated in this article, or claim that may be made by its manufacturer, is not guaranteed or endorsed by the publisher.
